The article "HBV Promotes the Proliferation of Liver Cancer Cells through the hsa_circ_0000847/miR-135a Pathway" was published in 2022. Journal: Evid Based Complement Alternat Med.

# HBV Promotes the Proliferation of Liver Cancer Cells through the hsa_circ_0000847/miR-135a Pathway

**DOI:** 10.1155/2022/7332337

**Published:** 2022-09-15

**Authors:** Jianjun Lin, Xiang Lian, Shihang Xue, Lian Ouyang, Lihui Zhou, Yuyang Lu, Longteng Xie

**Affiliations:** ^1^Department of Clinical Laboratory, Xiangshan First People's Hospital, Ningbo Fourth Hospital, Ningbo 315700, China; ^2^Hepatology Department, Xiangshan First People's Hospital, Ningbo Fourth Hospital, Ningbo 315700, China; ^3^Department of General Surgery, Xiangshan First People's Hospital, Ningbo Fourth Hospital, Ningbo 315700, China; ^4^Department of Orthopaedic Surgery, Xiangshan First People's Hospital, Ningbo Fourth Hospital, Ningbo 315700, China; ^5^Xiangshan County Center for Disease Control and Prevention, Ningbo 315700, China

## Abstract

Hepatocellular carcinoma (HCC) is currently one of the most common tumors, with a high morbidity and mortality rate. HCC induced by persistent hepatitis *B* virus (HBV) infection is the most common liver cancer subtype at present, and HBV-related HCC is highly malignant and its development mechanism still needs to be explored in depth. This study aimed to explore the molecular mechanism of hsa_circ_0000847 targeting miR-135a-5p (miR-135a) to regulate the proliferation, invasion, and apoptosis of liver cancer cells. The study found that the expression level of hsa_circ_0000847 in liver cancer tissues and cells was significantly increased, while the expression level of miR-135a was significantly decreased. Hsa_circ_0000847 promoted the proliferation of liver cancer cells and elevated the expression of the proliferation-related protein. In addition, hsa_circ_0000847 could promote the invasion of HBV-infected liver cancer cells and inhibit the cell apoptosis of liver cancer cells. At the same time, it significantly promoted the expression of antiapoptotic proteins and inhibited the expression of proapoptotic protein. Interestingly, the dual luciferase experiment proved that hsa_circ_0000847 directly targeted miR-135a. On the other hand, the combined effect of hsa_circ_0000847 and miR-135a further illustrated the effect of hsa_circ_0000847 on the proliferation, invasion, and apoptosis of liver cancer cells. In addition, further experiments have also found that HBV could promote the expression of p-p38, p-ERK, and p-JNK through the hsa_circ_0000847/miR-135a axis, thereby further activating the MAPK pathway. In short, HBV promotes the proliferation and invasion of liver cancer cells and inhibits apoptosis by regulating the hsa_circ_0000847/miR-135a pathway, which provided a theoretical basis for effective treatment of HBV-infected liver cancers.

## 1. Introduction

Hepatocellular carcinoma (HCC) is currently one of the most common malignant tumors, with a high incidence and fatality rate worldwide [1]. Although liver transplantation and surgical treatment have obtained good results as the first-line treatment of liver cancers, the clinical data show that the 5-year survival rate of patients with liver cancers is still not high [2]. The main reason is that liver cancers exert a markedly high survival rate, high degree of malignancy, rapid growth and proliferation ability, and high metastasis rate [3]. Therefore, a better understanding of the molecular mechanism of the growth and metastasis of liver cancer cells is essential for the treatment of HCC. Studies have pointed out that the loss of control of tumor cell growth and the malignant proliferation of tumor cells is an important reason for the malignant development of tumors [4]. On the one hand, the malignant proliferation of tumor cells may lead to the activation of oncogenes, which accelerates the cell cycle process [5]. On the other hand, the cell apoptosis might be inhibited and the cell gains “immortality,” so that it loses control and proliferates malignantly [6]. In addition to the malignant proliferation, tumor metastasis is also an important cause of cancer death [7]. The main cause of metastasis is the acquisition of tumor cell migration and invasion capability. The occurrence and development of liver cancer is an extremely complex process, which is triggered by many factors. Among them, hepatitis *B* virus (HBV) is an important cause of hepatocellular carcinoma. About 80% of liver cancers are caused by HBV infection [8]. Recent studies have shown that the viral protein of HBV itself can promote the malignant development of liver cancer by promoting the malignant proliferation and distant metastasis of tumor cells. For example, in HBV-related HCC, HBV's genomic product preS2 protein can enhance the proliferation of liver cancer cells [9]. HBV *X* protein, that is, HBV promotes the migration and invasion of liver cancer cells by upregulating the expression of FoxM1, causing liver cancer metastasis, ultimately leading to a poor prognosis [10].

Circular RNAs (circRNAs) are a type of endogenous noncoding RNAs with a closed circular structure, which are mainly produced by the variable shearing process of precursor RNAs (pre-mRNAs) [11]. CircRNAs are widely present in all eukaryotes and are very stable. Studies have found that circRNA occupies a considerable proportion of transcripts, and some expression abundance is even significantly higher than other transcripts. At the same time, circRNAs exert an important regulatory effect on gene expression and play an important biological function in the development of organisms, such as acting as a miRNA sponges, endogenous RNAs, and biomarkers [12]. circRNAs also play an important role in the diagnosis and treatment of diseases. Studies have found that circRNAs play an important role in the occurrence of some diseases, including arteriosclerosis, nervous system disorders, diabetes, and cancer. miRNA sponge is the most frequently reported roles of circRNA in many tumors [13–16]. Many RNA transcripts share binding sites with miRNAs, and they compete with each other to act as competitive endogenous RNAs (ceRNAs) to further regulate tumor development [17, 18]. For example, circHIPK3 sponge miR-558 can inhibit the expression of heparanase in bladder cancer cells [19]. In addition, the circular RNA profile of circPVT1 identified it as a proliferation factor and prognostic marker of gastric cancer, and circular RNAMTO1 was used as a sponge of miR-9 to inhibit the progression of hepatocellular carcinoma [20].

In the previous experiment, the differentially expressed circRNAs in HBV-infected liver cancer cells were screened by high-throughput sequencing, and the present study found that hsa_circ_0000847 was significantly highly expressed in liver cancer tissues and cells. Therefore, the study aims to explore the specific mechanism of hsa_circ_0000847 in HBV infection of liver cancer cells.

## 2. Methods

### 2.1. Clinical Samples

HBV-positive liver cancer specimens (*n* = 10) and HBV-negative liver cancer specimens (*n* = 10) were collected from HCC patients who underwent hepatectomy at Xiangshan First People's Hospital. The pathological diagnosis has been confirmed, and the patients have not received chemotherapy or radiotherapy. All the patients have written the consent for approval of the application of clinical samples for basic research, and this study was approved by the research medical ethics committee at the hospital.

### 2.2. Cell Culture

Human normal hepatocytes (LO2), liver cancer cells (Bel-7402, Huh7, and HepG2), and HepG2.2.15 (HBV-infected liver cancer cells) were cultured in Dulbecco's Modified Eagle Medium (DMEM) containing 10% fetal bovine serum (FBS) and 1% penicillin, and streptomycin at 37°C in a 5% CO_2_ incubator. When the degree of cell association reached 80%–90%, the cells were passed into next passage at a ratio of 1 : 2 to 1 : 3.

### 2.3. CCK-8 Assay

The cells were seeded at a density of 1 × 10^5^ cells/mL in a 96-well plate, and the five replicate groups were set up for each group. The experiments were performed according to the experimental requirements as previously described [21]. After the treatment, the DMEM medium containing 10% CCK-8 was added. 1–4 h later, a microplate reader was used to detect the absorbance (OD value) at a wavelength of 450 nm. The proliferation capacity of the cell was directly proportional to the absorbance of the cells.

### 2.4. Real-Time Quantitative PCR (RT-qPCR)

The TRIzol reagent was used to extract total RNAs from the tissues and cells as previously described [22]. According to the instructions, 1000 ng of total RNA was reversed and recorded into cDNAs. Then, the cDNAs were used as a template to perform the fluorescence quantitative PCR reaction of the target genes according to the SYBR Green *I* method. The design and synthesis of primers were obtained from Shanghai Sanitary Industry Co., Ltd., using *β*-actin or U6 as the internal reference. The 2^−ΔΔCT^ method was used to analyze the relative expression level of the target gene.

### 2.5. Western Blotting

The protein lysate was used to extract the total proteins in the cells, and the extracted proteins were quantified by the BCA method [23, 24]. In each group, samples of the same concentration of protein were subjected to SDS-PAGE electrophoresis; then, the protein was electrotransferred to the PVDF membrane. The 5% skimmed milk powder was used to block for 1 h at room temperature and the primary antibody was incubated overnight at 4°C and washed 3 times with PBST. Then, the HRP-labeled secondary antibody was incubated for 1 hour at room temperature. After washing with PBST 3 times, the expression of proteins was analyzed by the ECL chemiluminescence method.

### 2.6. Transwell Assay

The experiments were carried out according to the previous study [25]. Briefly, the cells were cultured in a serum-free medium for 24 h, and the concentration was adjusted to 5 × 10^5^/mL. Then, 100 *μ*L cells were seeded into the polycarbonate membrane in the upper chamber of the small chamber and 600 *μ*L of the serum-containing culture medium were added to the lower chamber. The cells were placed in a 37°C, 5% CO_2_ cell culture incubator for 24 h and then removed. The cells were carefully wiped off the lower surface of the polycarbonate membrane of the upper chamber with a cotton swab, fixed with methanol, stained with crystal violet, and the number of invaded cells were observed under a microscope.

### 2.7. Double Fluorescein Enzyme Report Assay

The miR-135a mimics or its negative control (miR-135a mimics NC) was co-transfected with the luciferase reporter vector WT-hsa_circ_0000847 or MUT-hsa_circ_0000847 into HEK293T cells, respectively; miR-135a mimics NC and WT-hsa_circ_0000847 co-transfection, miR-135a mimics and WT-hsa_circ_0000847 co-transfection, miR-135a mimics NC and mut-hsa_circ_0000847 co-transfection, and miR-135a mimics and MUT-hsa_circ_0000847 co-transfection. After 24 h of transfection, the cells were collected and the relative luciferase activity was detected by the dual luciferase reporter gene detection system.

### 2.8. Flow Cytometry Assay

Cell transfection was carried out according to the experimental requirements. After 24 h of transfection, the culture medium was discarded. The cells were washed twice with 1×PBS and discarded. The cells were digested with 0.3% trypsin without EDTA and collected. The cells were centrifuged at 2000 rpm at room temperature for 5 min, and then the supernatant was discarded and 1 ml 1 × PBS was added to resuspend the cells. The cells were centrifuged at 2000 rpm for 5 min at room temperature, and then the supernatant was discarded. The cells were resuspended in 300 *μ*L 1×binding buffer and 5 *μ*L AnnexinV-FITC was added in a dark room for 10 min. Then, 5 *μ*L PI solution was added in a dark room for 5 min. Then, 200 *μ*L 1 × binding buffer was added, and flow detection was performed within 1 h.

### 2.9. Statistical Analysis

The data were analyzed using the SPSS 20.0 statistical package (IBM, USA). The results of this study were expressed as means ± standard deviation. The comparisons among multiple groups were performed using one-way analysis of variance (ANOVA) followed by post-hoc test for multiple comparisons. *P* < 0.05 indicated a significant difference.

## 3. Results

### 3.1. The Expression of hsa_circ_0000847 and miR-135a in Liver Cancer Cells and Tissues

In order to explore the expression of hsa_circ_0000847 in liver cancers, we detected the expression levels of hsa_circ_0000847 and miR-135a in liver cancer cells and HBV-infected liver cancer cells. The results showed that the expression level of hsa_circ_0000847 in liver cancer cells was significantly higher than that of normal liver cells, especially in HBV-infected liver cancer cells (Figure 1(a)). While the expression level of miR-135a was significantly lower in liver cancer cells than that of normal liver cells, especially in HBV-infected liver cancer cells (Figure 1(b)). In addition, compared with HBV-negative liver cancer specimens, the expression level of hsa_circ_0000847 was significantly increased in HBV-positive liver cancer specimens, while the expression level of miR-135a was significantly decreased (Figures 1(c) and 1(d)). The results suggested that hsa_circ_0000847 and miR-135a might be related to the development and occurrence of liver cancer.

### 3.2. The Effects of hsa_circ_0000847 on the Cell Proliferation of Liver Cancer Cells

This study explored the effects of hsa_circ_0000847 on the cell proliferation through CCK-8 assay and detecting the expression of proliferation-related proteins. Compared with the HepG2 group, the OD values of the cells in pHBV1.3 + HepG2 group were markedly increased, which were reduced by pHBV1.3 + si-hsa_circ_0000847 + HepG2 (Figure 2(a)). Compared with the HepG2 group, the OD values of the cells were obviously decreased in si-hsa_circ_0000847 + HepG2 group (Figure 2(a)). Besides, the OD values of HepG2.2.15 group were inhibited by si-hsa_circ_0000847 + HepG2.2.15 (Figure 2(a)).

Furthermore, the results of western blot showed that the expression of proliferation-related proteins (PCNA and CyclinD1) was much higher in pHBV1.3 + HepG2 group than that in HepG2 group, which was reduced by si-hsa_circ_0000847+HepG2 (Figures 2(b)–2(d)). Furthermore, the expression of proliferation-related proteins (PCNA and CyclinD1) in si-hsa_circ_0000847 + HepG2.2.15 group was much lower than that in HepG2.2.15 group (Figures 2(b)–2(d)). The results indicated that HBV promoted the proliferation of liver cancer cells through hsa_circ_0000847.

### 3.3. The Effects of hsa_circ_0000847 on the Invasion of Liver Cancer Cells

To further analyze the effects of hsa_circ_0000847 on the invasion of liver cancer cells, the transwell experiments were carried out. The results showed that compared with the HepG2 group, the number of invasive cells in pHBV1.3 + HepG2 group was markedly increased, which were inhibited by pHBV1.3 + si-hsa_circ_0000847 + HepG2 (Figure 3). Compared with the HepG2 group, the number of invasive cells in HepG2.2.15 group was significantly increased, which was blocked by si-hsa_circ_0000847 + HepG2.2.15 (Figure 3). The results suggested that the number of cells in the si-circRNA group was significantly lower than that in the untransfected si-circRNA group (Figure 3). Therefore, hsa_circ_0000847 and HBV significantly enhanced the invasion ability of liver cancer cells.

### 3.4. The Effects of hsa_circ_0000847 on the Cell Apoptosis of Liver Cancer Cells

In addition, the experiments were applied to detect the effects of hsa_circ_0000847 in the apoptosis of liver cancer cells by flow cytometry and western blotting. The results showed that compared with the HepG2 group, the apoptosis rate of liver cancer cells in pHBV1.3 + HepG2 group was much lower, which was elevated by si-hsa_circ_0000847 (Figure 4(a)). Moreover, compared with HepG2.2.15 group, the apoptosis rate of liver cancer cells in si-hsa_circ_0000847 + HepG2.2.15 group was significantly increased (Figure 2(a)).

In addition, western blotting experiments also proved the results. The results of western blotting showed that compared with the HepG2 group, the apoptosis-related proteins (Bax and cleaved caspase-2) of liver cancer cells in pHBV1.3 + HepG2 group was much lower, which was upregulated by si-hsa_circ_0000847 (Figures 4(b)–4(c)). While the antiapoptosis-related protein Bcl-2 of liver cancer cells in pHBV1.3 + HepG2 group was much higher, which was decreased by si-hsa_circ_0000847 (Figures 4(b)–4(c)). Moreover, compared with the HepG2.2.15 group, the expression of Bax and cleaved caspase-2 of liver cancer cells in si-hsa_circ_0000847 + HepG2.2.15 group was significantly increased, while the expression of Bcl-2 was decreased (Figures 4(b)––4(c)). The results suggested that knockdown of hsa_circ_0000847 could significantly promote the apoptosis of liver cancer cells. In short, hsa_circ_0000847 exerted a significant antiapoptotic effect on liver cancer cells.

### 3.5. Targeting Relationship between hsa_circ_0000847 and miR-135a

Through the dual luciferase experiment, we found that the luciferase activity of the miR-135a mimics + MUT-hsa_circ_0000847 group was significantly lower than that of the MUT-hsa_circ_0000847 and miR-135a mimics NC co-transfection group (Figure 5). However, compared with the MUT-hsa_circ_0000847 and mimics NC co-transfection group, the luciferase activity of the MUT-hsa_circ_0000847 + miR-135a mimics group did not change significantly (Figure 5). The results suggested that hsa_circ_0000847 might directly target miR-135a.

### 3.6. The Effect of hsa_circ_0000847 and miR-135a on Cell Proliferation of Liver Cancer Cells

The cell proliferation experiments found that si-hsa_circ_0000847 + miR-135a-5p mimics can significantly inhibit the proliferation of liver cancer cells in the HepG2 + pHBV1.3 cell group (Figure 6(a)). Similarly, the HepG2.2.15 cell group has similar results, and the ability to inhibit the proliferation of liver cancer cells is stronger (Figure 6(b)). In addition, in HepG2.2.15 cells or HepG2 transfected with pHBV1.3, the miR-135a mimics + si-hsa_circ_0000847 group significantly reduced the expression levels of proliferation-related proteins PCNA and CyclinD1 (Figures 6(c) and 6(d)). All these results indicated that HBV promoted the proliferation of liver cancer cells through the hsa_circ_0000847/miR-135a axis.

### 3.7. The Effects of hsa_circ_0000847 + miR-135a on Cell Invasion of Liver Cancer Cells

Experiments have proved that hsa_circ_0000847 can promote the invasion ability of liver cancer cells. Therefore, the next step is to test the effects of si-circRNA + miR-135a on cell invasion of liver cancer cells. After experiment silencing hsa_circ_0000847, it was found that in the HepG2+pHBV1.3 cell group, miR-135a-5p mimics can significantly inhibit the invasion ability of liver cancer cells (Figure 7). Similarly, in the HepG2.2.15 cell group, miR-135a mimics also significantly inhibited the invasion of liver cancer cells (Figure 7). Therefore, whether in liver cancer cells or HBV-infected liver cancer cells, si-hsa_circ_0000847 can inhibit the invasion of liver cancer cells through miR-135a. Therefore, si-hsa_circ_0000847 + miR-135a can significantly inhibit the invasion of liver cancer cells.

### 3.8. The Effect of hsa_circ_0000847 + miR-135a on Cell Apoptosis of Liver Cancer Cells

In the HepG2.2.15 group, the co-transfection of miR-135a mimics and si-hsa_circ_0000847 significantly promoted the apoptosis of liver cancer cells (Figure 8(a)). At the same time, it elevated the expression level of the proapoptotic protein Bcl-2 and cleaved caspase-3 but inhibited the expression level of the protein Bax (Figure 8(b)). Importantly, the HepG2+pHBV1.3 group also got the same result (Figures 8(c) and 8(d)). The abovementioned results indicated that co-transfection of miR-135a mimics and si-hsa_circ_0000847 promoted the apoptosis of liver cancer cells.

### 3.9. The Effect of hsa_circ_0000847 + miR-135a on the Activation of the MAPK Pathway

The MAPK pathway plays an important role in the occurrence and development of cancers. In this study, compared with the control group, the si-hsa_circ_0000847 + miR-135a mimics group significantly reduces the expression levels of phosphorylated proteins p-p38, p-ERK, and p-JNK in HepG2.2.15 cells (Figure 9(a)). In HepG2 cells transfected with pHBV1.3, the expression levels of p-p38, p-ERK, and p-JNK were also significantly inhibited by miR-135a/ hsa_circ_0000847 (Figure 9(b)). Therefore, the findings showed that miR-135a/hsa_circ_0000847 will significantly inhibit the activation of the MAPK pathway.

## 4. Discussion

The development of liver cancer is a multistep process involving multiple genetic and epigenetic changes. Several studies have confirmed that dysregulated circRNAs are related to the progression of liver cancer. It is reported that the downregulation of hsa_circ_0001445 expression is significantly related to the aggressiveness of liver cancer, and it can be used as an independent risk factor for overall survival and recurrence-free survival of patients after hepatectomy [26]. Overexpression of hsa_circ_0001445 exerts an inhibitory effect on the proliferation and migration of liver cancer cells [26]. It has found that knockdown of circRNAs significantly inhibited the proliferation, cycle progression, and migration of liver cancer cells [27]. Therefore, restoring the expression of liver cancer-related circRNAs might exert an inhibitory effect on the progression of liver cancer. In our study, the expression of hsa_circ_0000847 in liver cancer tissues was significantly increased, suggesting that the dysregulated expression in hsa_circ_0000847 might be related to the progression of liver cancer. Besides, the knockdown of hsa_circ_0000847 significantly reduces the viability of liver cancer cells HepG2 and HepG2.2.15, suggesting that hsa_circ_0000847 exerted a pro-proliferation effect in liver cancer cells.

As we all know, Bax, Bcl-2, and cleaved caspase-3 proteins play an important role in the apoptosis of tumor cells, and their abnormal expression is critical to the occurrence and development of cancer [24, 28, 29]. This study showed that knockdown of hsa_circ_0000847 significantly increased the expression of Bax and cleaved caspase-3 proteins, and decreased the expression of Bcl-2 protein. In addition, the MAPK pathway is a classic inflammation and tumor-related pathway, which plays an important role in the regulation of liver cancer. The previous studies have shown that circ-MAPK4 inhibits glioma cell apoptosis through the MAPK signaling pathway by secreting miR-125a-3p [30]. circ_0001721 promotes the progression of osteosarcoma through the miR-372-3p/MAPK7 axis [31]. Therefore, to explore the effects of hsa_circ_0000847 on liver cancers, it is necessary to focus on the roles of MAPK pathway. In this study, si-hsa_circ_0000847 significantly inhibited the expression levels of p-p38, p-ERK1/2, and p-JNK1/2/3 in HepG2.2.15 cells. Therefore, hsa_circ_0000847 participates in the regulation of liver cancer cells by activating the MAPK pathway.

miRNA is an endogenous noncoding small RNA consisting of about 22 nucleotides and is an essential epigenetic regulatory factor in cancer [32–34]. A number of studies have shown that circRNAs can directly interact with miRNAs to regulate the expression of target genes and participate in the progression of liver cancers [35–37]. For example, circMAT2B promotes glycolysis of liver cancer cells by regulating the miR-338-3p/PKM2 axis under hypoxic conditions, thereby promoting liver cancer progression [38]. miR-21 is involved in cellular processes, such as cell proliferation, angiogenesis, invasion, and metastasis, and resistance to chemotherapy and radiotherapy. It is a carcinogenic factor for breast cancer and non-small cell lung cancers [39, 40]. The high expression of miR-21 in liver cancer is associated with shortened 5-year overall survival and 5-year disease-free survival of liver cancer patients, which suggests miE-21 is a potential prognostic marker of liver cancer [41]. This study confirmed that miR-135a binds directly and specifically to circRNAs, and the expression of miR-135a is negatively regulated by circRNAs. Analysis of the function of miR-135a showed that inhibiting the expression of miR-135a significantly downregulated the expression of Bcl-2 protein, upregulated expression of Bax, and cleaved caspase-3 proteins, and inhibited the proliferation and invasion of HepG2.2.15 cells.

In summary, the expression of hsa_circ_0000847 in liver cancer tissues is upregulated. The knockdown of hsa_circ_0000847 can reduce the proliferation and invasion of liver cancer cells and its mechanism is related to the negative regulation of miR-135a expression. This provides new clues for understanding the role of circRNAs/miRNAs regulatory network in liver cancer and provides a valuable target for liver cancer treatment.

## Figures and Tables

**Figure 1:** The expression level of hsa_circ_0000847/miR-135a in liver cancer cells. (a and b) Elevated expression of hsa_circ_0000847 and decreased expression of miR-135a in liver cancer cell lines (*n* = 3, mean ± SD, ^*∗*^*p* < 0.05, ^*∗∗*^*p* < 0.01, ^*∗∗∗*^*p* < 0.001 vs LO2 cells). (c and d) Elevated expression of hsa_circ_0000847 and decreased level of miR-135a in HBV-positive liver cancer specimens (*n* = 10, mean ± SD, ^*∗*^*p* < 0.05, ^*∗∗*^*p* < 0.01, ^*∗∗∗*^*p* < 0.001 vs HBV-negative liver cancer specimens).

**Figure 2:** The effects of si-hsa_circ_0000847 on cell proliferation and the protein expression of PCNA and CyclinD1. (a) si-circRNA reduced the proliferation of HepG2, pHBV1.3 + HepG2, and HepG2.2.15 cells. (b-d) si-circRNA reduces the protein expression of PCNA and CyclinD1 (*n* = 3, Mean ± SD, ^*∗*^*p* < 0.05, ^*∗∗*^*p* < 0.01, ^*∗∗∗*^*p* < 0.001.

**Figure 3:** The effects of si-hsa_circ_0000847 on cell invasion. Transwell assay was applied to detect the invasion ability of liver cancer cells (*n* = 3).

**Figure 4:** The effect of si-hsa_circ_0000847 on cell apoptosis in liver cancer cells. (a). Flow cytometry was used to detect the effect on cell apoptosis. (b and c) The expression levels of apoptosis-related proteins Bcl-2, Bad, and cleaved caspase-3 (*n* = 3, Mean ± SD, ^*∗∗*^*p* < 0.01, ^*∗∗∗*^*p* < 0.001.

**Figure 5:** The relationship between hsa_circ_0000847 and miR-135a. Double luciferase reporter gene assay was performed in 293T cells, and the ratio of firefly/Renilla activity represents luciferase activity (*n* = 3, mean ± SD, ^*∗*^*p* < 0.5.

**Figure 6:** The effects of si-circRNA on cell proliferation and the protein expression of PCNA and CyclinD1. (a and b) The proliferation of HepG2 + pHBV1.3 cells (a) and HepG2.2.15 cell group (b) tested by CCK-8. (c and d) The expression levels of apoptosis-related proteins PCNA and CyclinD1 in HepG2 + pHBV1.3 cell group (c) and HepG2.2.15 cell group (d). *n* = 3, Mean ± SD, ^*∗*^*p* < 0.05, ^*∗∗*^*p* < 0.01, ^*∗∗∗*^*p* < 0.001 vs control.

**Figure 7:** The effects of si-hsa_circ_0000847 and miR-135a on cell invasion. The effects of miR-135a-5p, mimics si-hsa_circ_0000847, and miR-135a-5p mimics + si-hsa_circ_0000847 on cell invasion in HepG2 + pHBV1.3 and HepG2.2.15 groups, respectively (*n* = 3).

**Figure 8:** The roles of si-hsa_circ_0000847 and miR-135a on cell apoptosis. (a) Flow cytometry was used to detect cell apoptosis in HepG2.2.15 cells. (b) The expression levels of apoptosis-related proteins Bcl-2, Bad, and cleaved caspase-3 in HepG2.2.15 cells. (c) Flow cytometry was used to detect cell apoptosis in HepG2+pHBV1.3 cells. (d) The expression levels of apoptosis-related proteins Bcl-2, Bad, and cleaved caspase-3 in HepG2 + pHBV1.3 cells. *n* = 3, mean ± SD, ^*∗*^*p* < 0.05, ^*∗∗*^*p* < 0.01, ^*∗∗∗*^*p* < 0.001 vs control.

**Figure 9:** The roles of si-hsa_circ_0000847 and miR-135a on the activation of MAPK pathway. (a and b) The expression levels of p-ERK, ERK, p-JNK, JNK, p-p38, and p38 in the HepG2.2.15 group (a) and the HepG2 + pHBV1.3 group (b).

## Data Availability

All data included in this study are available upon request by contacting the corresponding author.
